# MircoRNA‐1275 promotes proliferation, invasion and migration of glioma cells via SERPINE1

**DOI:** 10.1111/jcmm.13760

**Published:** 2018-07-19

**Authors:** Dong‐Mei Wu, Shan Wang, Xin Wen, Xin‐Rui Han, Yong‐Jian Wang, Shao‐Hua Fan, Zi‐Feng Zhang, Qun Shan, Jun Lu, Yuan‐Lin Zheng

**Affiliations:** ^1^ Key Laboratory for Biotechnology on Medicinal Plants of Jiangsu Province School of Life Science Jiangsu Normal University Xuzhou China; ^2^ College of Health Sciences Jiangsu Normal University Xuzhou Jiangsu China

**Keywords:** glioma, MiR‐1275, p53 signalling pathway, SERPINE1

## Abstract

This study was designed to explore the relationship between miR‐1275 and SERPINE1 and its effects on glioma cell proliferation, migration, invasion and apoptosis. Differentially expressed miRNAs and mRNAs in glioma tissues were screened out by bioinformatic analysis. Dual‐luciferase reporter gene assay was used to validate the targeted relationship between miR‐1275 and SERPINE1. qRT‐PCR was used to detect the expression of miR‐1275 and SERPINE1 in glioma tissues. The expressions of SERPINE1 and p53 pathway‐related proteins in glioma cells were detected by western blot. Glioma cell proliferation, apoptosis, migration and invasion were respectively detected by CCK‐8 assay, flow cytometry, wound healing assay and transwell assay. Tumour xenograft model was developed to study the influence of miR‐1275 and SERPINE1 on glioma growth in vivo. The results of microarray analysis, qRT‐PCR and western blot showed that miR‐1275 was low‐expressed while SERPINE1 was high‐expressed in glioma. Dual‐luciferase assay showed that miR‐1275 could bind to SERPINE1. Overexpression of miR‐1275 could promote the p53 pathway‐related proteins’ expression. Highly expressed miR‐1275 could repress the migration, proliferation and invasion of glioma cells while highly expressed SERPINE1 had inverse effects. Tumour xenograft showed that up‐regulated miR‐1275 or down‐regulated SERPINE1 could repress glioma growth in vivo. Up‐regulation of miR‐1275 activated p53 signalling pathway via regulating SERPINE1 and therefore suppressed glioma cell proliferation, invasion and migration, whereas promoted cell apoptosis.

## 1 INTRODUCTION

Glioma, a kind of malignancy arising from glial cells in the brain, is the most common malignant tumours occurring in the central nervous system and accounting for 78% of intracranial primary tumours.^1^, ^2^ Glioma usually exhibits a series of malignant features, including extensive, rapid and aggressive progression, resistance to surgery, radiotherapy and chemotherapy, all of which lead to the poor prognosis for most patients.^3^ Although extensive efforts have been made to improve glioma treatment, average survival time of the patients remains 11‐15 months.^4^ Consequently, it is imperative to further explore the pathogenesis of glioma and discern potential biomarkers.

MicroRNAs (miRNAs) are small non‐coding RNA molecules with a length of about 16‐24 nucleotides.^5^ It is generally considered that miRNAs exert their activities at the post‐transcriptional level. They can bind to 3′ untranslated regions (3′UTR) of the mRNAs transcribed from their target genes, and therefore led to mRNA degradation or repression of protein translation.^6^ The dysregulation of miRNAs has been confirmed to be strongly related with tumorigenesis, and miRNAs work as tumour promoters or suppressors due to regulation of different target genes.^7^ Glioma is no exception. Increasing evidences suggest that various miRNAs are aberrantly expressed in glioma.^8^ To further study the effects of differential expressed miRNAs in glioma, we performed bioinformatic analysis and put our eyesight on an aberrantly low‐expressed miRNA miR‐1275. MiR‐1275 has been reported to influence multiple diseases, such as inhibiting adipogenesis in obese,^9^ repressing tumour growth of hepatocellular carcinoma^10^ as well as influencing oligodendroglial differentiation of glioma stem‐like cells.^11^ Herein, we explored the specific mechanism of miR‐1275 on targeting its target genes in glioma, which had not been studied before.

P53 signalling pathway reported as the “guardian of the genome” functions at the centre of a complex molecular network to mediate tumour suppression. It is essential for p53‐mediated cell signal transduction pathway to regulate the normal life activities of cells.^12^ Numerous studies have shown that p53 signalling pathway is closely linked to tumorigenesis. P53 has been known to mutate in more than 50% of human cancers,^13^ including glioma. A previous study found that p53 signalling pathway was found to be dysregulated in 85.3% of glioma patients according to the TCGA (The Cancer Genome Atlas) data.^14^ Herein, we analysed signalling pathways closely related to glioma using Gene Set Enrichment Analysis (GSEA) to confirm the aberrant condition of p53 pathway. Moreover, based on Kyoto Encyclopedia of Genes and Genomes (KEGG) dataset, we found that a member of p53 signalling pathway, SERPINE1, was predicted to have the targeting relationship with miR‐1275, reminding that miR‐1275 might exert its function through p53‐related genes.

SERPINE1, also called plasminogen activator inhibitor type 1 (PAI‐1), works as the inhibitor of tissue plasminogen activator (tPA) as well as urokinase (uPA), and hence is a fibrinolysis inhibitor. Many previous studies have detected its aberrant expression in cancers. For instance, SERPINE1 was found to be high‐expressed in colorectal cancer and related to tumour invasiveness and aggressiveness.^15^ Overexpression of SERPINE1 has also been found in many other cancers including melanoma,^16^ oesophageal cancer^17^ and bladder cancer.^18^ It can be seen as a poor prognosis biomarker. Parallelly, bioinformatic analysis on glioma conducted by us also found that SERPINE1 was high‐expressed and related with patients’ prognosis.

Thus, our study was performed to investigate the effects of miR‐1275 on repressing p53‐related gene SERPINE1 and therefore influencing the biological functions of glioma cells, including proliferation, apoptosis, migration and invasion. Our discovery might contribute to perceiving the in‐depth molecular mechanism of glioma tumorigenesis.

## 2 MATERIALS AND METHODS

### 2.1 Clinical samples

Clinical glioma tissues were collected from 30 glioma patients that underwent glioma resection at Key Laboratory for Biotechnology on Medicinal Plants of Jiangsu Province, School of Life Science, Jiangsu Normal University from September 2011 to October 2014. Normal brain tissues were collected from 11 patients who died of glioma and 19 patients died of other diseases. For glioma patients, normal tissues were taken from the brain tissues more than 3 cm from the border of the glioma tissues. All specimens were supported by Medical Ethics Committee of Key Laboratory for Biotechnology on Medicinal Plants of Jiangsu Province, School of Life Science, Jiangsu Normal University and all patients and their family members had signed the informed consents. Tissue specimens were taken immediately after the material and stored at −80°C.

### 2.2 Bioinformatic analysis

Clinical information about glioma (5 normal brain tissues and 5 primary glioma tissues) was obtained from TCGA database (The Cancer Genome Atlas, https://cancergenome.nih.gov). Differentially expressed miRNAs and mRNAs were filtered using Bioconductor R version 3.4.1 (https://www.r-project.org/) and “Limma” program package. The screening thresholds were | log_2_(fold change) | >2 and adjusted *P* value <.05. Based on the analysis results of differentially expressed mRNAs, the signalling pathways closely related to gliomas were analysed by GSEA (http://software.broadinstitute.org/gsea/msigdb/index.jsp) for subsequent studies.

### 2.3 Cell culture and transfection

Human normal glial cell line HEB, human glioma cell line U251, H4 and TJ905 were purchased from BeNa Culture Collection (Beijing, China). All the cells were cultured in Dulbecco's Modified Eagle Medium (DMEM; Gibco, Grand Island, NY, USA) containing 10% foetal bovine serum (FBS; Gibco) and preserved at 37°C with 5% CO_2_. MiR‐1275 mimics, control mimics and pcDNA3.1‐SERPNE1 plasmids were obtained from GenePharma (Shanghai, China). Above compounds were transfected into U251 cells using Lipofectamine 3000 reagent (Invitrogen, Carlsbad, CA, USA) respectively on the grounds of the manufacturer's protocol, and cells were collected for following experiments 48 hours after transfection.

### 2.4 qRT‐PCR

The total RNA was extracted with Trizol reagent (Invitrogen). RNA was reverse‐transcripted to cDNA using Super Script^™^ III Reverse Transcriptase Kit (Invitrogen) and TaqMan^™^ MicroRNA Reverse Transcription Kit (Applied Biosystems, Foster City, CA, USA). Quantitative PCR was then performed using SYBR^™^ Select Master Mix (Applied Biosystems) on LightCycler 480 PCR System (Roche, Rotkreuz, Switzerland) following the manufacture's protocol. U6 and β‐actin were respectively regarded as the internal reference for miRNA and mRNA. Relative expression of miR‐1275 and SERPINE1 was calculated using $2^{-\Delta \Delta C_{t}}$ method. All the reactions were repeated for 4 times. Primer sequences were listed in Table 1.

**Table 1:** qRT‐PCR primer sequence

Gene	Primer sequence
miR‐1275 forward	5′‐CGTGGGGGAGAGGCTGTC‐3′
U6 forward	5′‐CTCGCTTCGGCAGCACATA‐3′
U6 reverse	5′‐AACGATTCACGAATTTGCGT‐3′
SERPINE1 forward	5′‐CAGACCAAGAGCCTCTCCAC‐3′
SERPINE1 reverse	5′‐GGTTCCATCACTTGGCCCAT‐3′
β‐actin forward	5′‐CCGTTCCGAAAGTTGCCTTTT‐3′
β‐actin reverse	5′‐ATCATCCATGGTGAGCTGGC‐3′

### 2.5 Dual‐luciferase reporter gene assay

The binding site between miR‐1275 and SERPINE1 3′ untranslated regions (3′UTR) was predicted by TargetScan database version 7.1 (http://www.targetscan.org/vert_71). Wild‐type (wt) and mutant‐type (mut) SERPINE1 3′UTR were separately inserted into pMIR‐REPORT vectors (Ambion, Austin, TX, USA). Vectors and miR‐1275 mimics or negative control were co‐transfected into HEK‐293T cells, then luciferase activity was detected using Dual‐Luciferase Reporter Assay system (Promega, Madison, WI, USA).

### 2.6 Western blot

Total proteins were isolated using RIPA lysis buffer (Sigma‐Aldrich, St. Louis, MO, USA) and quantified using Bicinchoninic Acid (BCA) Kit (Sigma‐Aldrich). The obtained proteins were then separated by 12% SDS‐PAGE and transferred onto PVDF membranes (Invitrogen). The membranes were hindered in 5% nonfat milk for 1 hour, and incubated overnight with primary antibodies at 4°C, followed by secondary antibody HRP‐labelled goat anti‐rabbit IgG (1:2000, #ab6721; Abcam, Cambridge, MA, USA) for 1 hour at 37°C. After incubation, ECL Western Blotting Substrate Kit (Abcam) was used to detect immunoblots. Primary antibodies were as follows: rabbit anti‐p21 (1:1000, #ab109520; Abcam), rabbit anti‐Bax (1:1000, #ab32503; Abcam), rabbit anti‐Caspase3 (1:500, #ab13847; Abcam), rabbit anti‐cleaved Caspase3 (1:500, #ab32042; Abcam) and rabbit anti‐GAPDH (internal reference) (1:2500, #ab9485; Abcam).

### 2.7 CCK‐8 assay

CCK‐8 assay was performed to detect cell viabilities using Cell Counting Kit‐8 (Sigma‐Aldrich). Cells were seeded in 96‐well plates (2 × 10^3^ per well). After cultured for 1, 2, 3, 4 or 5 days, cells were incubated with10 μL CCK‐8 reagent for 4 hours at 37°C. The absorbance was detected at the wavelength of 450 nm on Multiskan^™^ GO microplate reader (Thermo Fisher Scientific, Waltham, MA, USA).

### 2.8 Flow cytometry assay

Apoptosis was detected using Apoptosis and Necrosis Assay Kit (Beyotime, Shanghai, China) according to the manufacturer's instruction. The glioma cells were harvested and washed twice with cold PBS. The cells were then successively stained with 5 μL Annexin V‐fluorescein isothiocyanate (FITC) and 5 μL Propidium Iodide (PI) solution, and subsequently incubated in a dark room for 15 minutes at room temperature. Flow cytometry was performed on FACSVerse^™^ flow cytometer (BD Biosciences, San Jose, CA, USA). Both early and late populations of apoptotic cells were calculated. The condition of gating set was based on the distribution of normal glioma cells (covering the accumulation area of non‐apoptotic cells).

### 2.9 Wound healing assay

Cells were sowed in 6‐well plates and cultured until they grew to a density of about 80%, then a wound was generated by manually scraping the cell monolayer with a 10 μL sterile pipette tip. Cells were washed by PBS and then cultured with fresh serum‐free medium at 37°C, 5% CO_2_. Cell migration was observed at 2 preselected time points (0 and 48 hours). Images of the scratches were filmed under the optical microscope.

### 2.10 Transwell invasion assay

Transwell invasion assay was performed in 24‐well cell culture chambers using transwell inserts (Corning Incorporated, Corning, NY, USA) with 8 μm pore size. The membranes of transwell inserts were coated with DMEM‐diluted Matrigel (BD Biosciences). 10^5^ cells were resuspended in 100 μL serum‐free medium and plated into upper chamber. DMEM with 10% FBS (500 μL/well) was added as chemoattractant in the lower chamber. After incubation for 8 hours, cells on upper surface of the insets were removed with a cotton swab, while cells on lower surface were immobilized with 4% paraformaldehyde for 15 minutes, air dried and then stained for 15 minutes with 0.1% crystal violet. Invasive cells were viewed and counted under the optical microscope.

### 2.11 Tumour xenograft

12 BALB/c (nu/nu) nude mice (aged 4‐6 weeks, weight 18‐24 g) were provided by the experimental animal centre of Key Laboratory for Biotechnology on Medicinal Plants of Jiangsu Province, School of Life Science, Jiangsu Normal University, and the in vivo experiment was approved by Medical Ethics Committee of Key Laboratory for Biotechnology on Medicinal Plants of Jiangsu Province, School of Life Science, Jiangsu Normal University. 100 μL cell suspension (containing 1.5 × 10^6^ U251 cells) was injected into the dorsal skin of each mice. After visible tumours were formed, mice were randomly divided into 3 groups (4 per group). Mice in the NC group were injected with 30 μL 10^8^TU/mL lentiviral control shRNA and 30 nmol control agomir, while those in Agomir‐1275 group were injected with 30 nmol agomir‐1275, and those in sh‐SERPINE1 group were injected with 30 μL 10^8^ TU/mL lentiviral sh‐SERPINE1. All the compounds were injected into tumour tissues per 2 weeks. Tumour volume was measured per 5 days with caliper and counted following the formula: V = [(length + width)/2]^3^ × 0.5236. All mice were sacrificed at 30th day, and tumour tissues were excised and weighed.

### 2.12 Immunohistochemistry

Mice tumour tissues were collected and made into 5‐μm paraffin‐embedded sections. Sections were dewaxed at 67°C, and then endogenous peroxidase was inactivated with 3% hydrogen peroxide methanol solution. Non‐specific antigens were blocked with 10% goat serum at 37°C for 1 hour. After washing thrice with PBS, sections were incubated at 37°C for 1.5 hours with primary antibodies, and then incubated with secondary antibody for 1 hour at room temperature. Then sections were washed with PBS and incubated with 3, 3′‐Diaminobenzidine (DAB; Sigma‐Aldrich) for 5 minutes in a dark room. After being washed with PBS, sections were then counterstained for 1 minute with hematoxylin (Sigma‐Aldrich). Permount^™^ Mounting Medium (Abcam) was utilized to mount the sections. Primary antibodies used were as listed below: rabbit anti‐SERPINE1 (5 μg/mL, ab66705; Abcam), rabbit anti‐p53 (20 μg/mL, ab1431; Abcam), rabbit anti‐MDM2 (1:100, ab131355; Abcam), rabbit anti‐cleaved Caspase3 (10 μg/mL, ab2302; Abcam) and rabbit anti‐ki67 (1:50, ab8191; Abcam). Secondary antibody was HRP‐labelled goat anti‐rabbit IgG (1:2000, ab205718; Abcam).

### 2.13 Statistical analysis

Graphpad Prism version 6.0 (GraphPad Software, La Jolla, CA, USA) was used to analyse the experimental data and the results were presented in form of mean ± standard deviation (SD). Comparison between the 2 sets of data was performed using Student's *t* test, and differences between the 3 or more groups of data were compared by one‐way ANOVA. All experiments were carried repeatedly for 4 times. *P* < .05 signified a statistical significance.

## 3 RESULTS

### 3.1 Bioinformatic analysis

Based on the RNA expression profiles of glioma patients from TCGA, we screened out differentially expressed miRNAs and mRNAs in glioma. Top‐30 differentially expressed miRNAs (Figure 1A) and mRNAs (Figure 1B) were shown in the heat maps (differentially expressed miRNAs and mRNAs were also listed in Table 2). Among those differential expressed RNAs, we selected low‐expressed miRNA miR‐1275 and high‐expressed mRNA SERPINE1, which have potential correlation (Figure 1C). Furthermore, GSEA analysis exhibited that p53 signalling pathway was down‐regulated according to the gene expression profile of glioma (Figure 1D), and SERPINE1 was involved in it. Prognostic analysis also showed that the overall survival rate of patients with SERPINE1 high‐expression was poorer (Figure 1E). Herein, we suggest that miR‐1275 might affect glioma cell function through binding to SERPINE1 and therefore regulate p53 signalling pathway.

**Figure 1:** Bioinformatic analysis (A) Heat map of top‐30 differentially expressed miRNAs in glioma, miR‐1275 was one of lowly expressed miRNAs. B, Heat map of top‐30 differentially expressed mRNAs in glioma, SERPINE1 was one of highly expressed mRNAs. C, Predicted binding site between miR‐1275 and SERPINE1 3′UTR. D, GSEA analysis result showed that p53 signalling pathway was down‐regulated in glioma. E, The OS curve of SERPINE1. Overall survival rate of patients with high SERPINE1 expression was poorer

**Table 2:** Top‐30 differentially expressed miRNAs and mRNAs

miRNA (up)	Log_2_FC	miRNA (down)	Log_2_FC	mRNA (up)	Log_2_FC	mRNA (down)	Log_2_FC
hsa‐mir‐10b	9.8869284	hsa‐mir‐7156	−3.242451	Sep‐14	13.399512	DDN	−6.5134769
hsa‐mir‐888	7.6505258	hsa‐mir‐1298	−3.3134633	HOXD13	10.820494	TRHDE	−6.5314219
hsa‐mir‐892b	6.9157403	hsa‐mir‐495	−3.3824816	HOXD10	10.331299	C1QL3	−6.5641224
hsa‐mir‐891a	6.5791038	hsa‐mir‐487b	−3.4199812	HOXC11	10.258605	LL0XNC0116G2.1	−6.6059649
hsa‐mir‐892a	6.4657298	hsa‐mir‐1229	−3.4277692	HOXC10	10.185768	TESPA1	−6.6059999
hsa‐mir‐891b	6.133674	hsa‐mir‐889	−3.4285187	HOXA3	10.178346	NWD2	−6.6416005
hsa‐mir‐4788	5.3686959	hsa‐mir‐329‐2	−3.4408148	HOXC13	10.092682	CCBE1	−6.6456952
hsa‐mir‐548f‐1	5.0521791	hsa‐mir‐432	−3.4808634	HOXA5	10.045187	DRD5	−6.6646477
hsa‐mir‐4697	5.0421241	hsa‐mir‐1197	−3.5335421	NKX2‐5	9.9961422	KCNG3	−6.6860522
hsa‐mir‐1275	4.8758923	hsa‐mir‐412	−3.5437495	PITX2	9.9913918	OPRM1	−6.7607132
hsa‐mir‐892c	4.7130225	hsa‐mir‐656	−3.5535832	HOXA4	9.8929685	PNMA5	−6.8477496
hsa‐mir‐183	4.6201642	hsa‐mir‐203b	−3.5579117	ADAMDEC1	9.6478632	TMEM132D	−6.8779312
hsa‐mir‐4760	4.5829882	hsa‐mir‐329‐1	−3.5758108	TBX5	9.5104643	HIPK4	−6.8981916
hsa‐mir‐639	4.2009872	hsa‐mir‐323b	−3.6167502	HOXA7	9.4640977	MC4R	−6.9242088
hsa‐mir‐182	4.1138902	hsa‐mir‐490	−3.6490338	GATA4	9.340126	GPR52	−6.9443586
hsa‐mir‐5091	3.7609697	hsa‐mir‐431	−3.7116129	HOXA10	9.2573154	GJB6	−6.9545281
hsa‐mir‐7706	3.7433915	hsa‐mir‐218‐2	−3.7777188	HOXB4	9.2340852	RYR2	−6.9877107
hsa‐mir‐3610	3.6571012	hsa‐mir‐323a	−3.7850225	HOXA6	8.8832565	MCHR2	−7.0137697
hsa‐mir‐3193	3.6251633	hsa‐mir‐218‐1	−3.789657	HOXA9	8.1017036	NEFM	−7.0170256
hsa‐mir‐6507	3.4108424	hsa‐mir‐1912	−3.8970888	HOXD9	8.0745049	CNGB1	−7.1313954
hsa‐mir‐4746	3.3159618	hsa‐mir‐4501	−3.9449579	FOXD3	7.7688666	WIF1	−7.1854484
hsa‐mir‐320c‐1	3.2732934	hsa‐mir‐137	−4.0207265	EN1	7.7241032	GSG1L2	−7.237351
hsa‐mir‐195	3.1987765	hsa‐mir‐668	−4.0811775	HOXC9	7.2952745	GRIN1	−7.3108912
hsa‐mir‐10a	3.1470934	hsa‐mir‐485	−4.1228788	SERPINE1	7.0295463	NPBWR1	−7.3201318
hsa‐mir‐135a‐1	3.1374324	hsa‐mir‐433	−4.1506626	SHOX2	6.6276443	SYT10	−7.4374763
hsa‐mir‐224	3.1312373	hsa‐mir‐1264	−4.4953867	HAND2	6.5481258	CARTPT	−7.5464153
hsa‐mir‐21	3.0742729	hsa‐mir‐873	−4.6301271	HOXD11	6.4988817	SLC22A9	−7.5489614
hsa‐mir‐3074	3.0695843	hsa‐mir‐770	−4.7271268	MNX1	6.4199838	GPR6	−7.7096791
hsa‐mir‐551b	2.8874113	hsa‐mir‐448	−5.0239703	HOXA11	6.3371303	KLK7	−9.0846482
hsa‐mir‐497	2.8189617	hsa‐mir‐876	−5.2363364	SLC18A3	6.1268565	SLC22A8	−9.4145632

### 3.2 MiR‐1275 was low‐expressed while SERPINE1 was high‐expressed in glioma

The expression of miR‐1275 in glioma tissue was obviously lower than that in adjacent tissues (*P* < .05, Figure 2A) while SERPINE1 was significantly highly expressed (*P* < .05, Figure 2B). Parallelly, the expression of miR‐1275 in glioma cell lines U251 and TJ905 was significantly less than in normal neurogliocyte HEB, and U251 had the lowest miR‐1275 expression (*P* < .01, Figure 2C). U251 also showed the highest proliferation ability among 3 cell lines (*P* < .01, Figure 2D). Therefore, U251 cell line was selected for subsequent experiments.

**Figure 2:** MiR‐1275 was low‐expressed in gliomas while SERPINE1 was high‐expressed in glioma. A, Expression of miR‐1275 in glioma tissues was higher than that in adjacent tissues. *P < .05, compared with adjacent tissues; (B) Expression of SERPINE1 in glioma tissues was significantly lower than that in adjacent tissues. *P < .05, compared with adjacent tissues; (C) The endogenous expression of miR‐1275 in glioma cell lines (U251 and TJ905) was higher than that in normal human glial cells (HEB). D, CCK‐8 assay detected the proliferation activity of human glioma cells and human normal glial cells. *P < .05, **P < .01, compared with HEB group

### 3.3 SERPINE1 was the target gene of miR‐1275

The binding sites between miR‐1275 and SERPINE1 3′UTR were predicted by TargetScan (Figure 3A) and confirmed by dual‐luciferase reporter gene assay. Luciferase activity did not remarkably change in SERPINE1 mut + miR‐1275 mimics group while it significantly decreased in SERPINE1 wt + miR‐1275 mimics group (*P* < .01, Figure 3B). Furthermore, the expressions of both SERPINE1 mRNA (*P* < .01, Figure 3C) and protein (*P* < .01, Figure 3D) were down‐regulated after miR‐1275 mimics transfection. All these results indicated that SERPINE1 was the target gene of miR‐1275.

**Figure 3:** SERPINE1 was the target gene of miR‐1275. A, The predicted binding site between MiR‐1275 and SERPINE1 3′UTR; (B) The results of dual‐luciferase reporter gene assay showed that luciferase activity significantly decreased after co‐transfection of miR‐1275 mimics and SERPINE1 wt 3′UTR, while miR‐1275 mimics + SERPINE1 mut 3′UTR had no changes. C, Expression of SERPINE1 in miR‐1275 mimics group was significantly lower than the NC group. D, Western blot: SERPINE1 protein expression in miR‐1275 mimics group was decreased. **P < .01, compared with the NC group

### 3.4 MiR‐1275 repressed proliferation, migration and invasion whereas promoted apoptosis of glioma cells

MiR‐1275 mimics and control mimics (NC) were respectively transferred into U251 cells and detected by qRT‐PCR. The result showed a remarkable increase in miR‐1275 expression after transfection (*P* < .001, Figure 4A). CCK‐8 assay showed that miR‐1275 mimics significantly reduced the proliferation ability of U251 cells (*P* < .01, Figure 4B). Flow cytometry revealed that cell apoptosis rate was remarkably increased after miR‐1275 mimics’ transfection (*P* < .01, Figure 4C). Migration and invasion of U251 cells with miR‐1275 mimics transfected were decreased according to the results of wound healing assay (*P* < .01, Figure 4D) as well as transwell migration assay (*P* < .01, Figure 4E). As a consequence, miR‐1275 could repress glioma cell proliferation, migration and invasion whereas promote cell apoptosis.

**Figure 4:** MiR‐1275 repressed proliferation, invasion and migration of glioma cells while induced its apoptosis. A, Relative expression of miR‐1275 in miR‐1275 mimics group was remarkably increased. B, Cell survival rate of miR‐1275 mimics group was higher than that of the NC group. C, Cell apoptosis rate in miR‐1275 mimics group was significantly higher than in the NC group. D, Closed wound area in miR‐1275 mimics group was less than that in the NC group. E, Number of invasive cells in miR‐1275 mimics group was significantly lower than that in the NC group. **P < .01, ***P < .001, compared with the NC group

### 3.5 MiR‐1275 represses glioma cell proliferation, migration and invasion whereas promotes cell apoptosis through targeting SERPINE1

Western blot was used to detect SERPINE1 expression in U251 cells after transfection. The result showed that SERPINE1 expression could be promoted by pcDNA3.1‐SERPINE1 while repressed by miR‐1275 mimics (*P* < .01, Figure 5A). Cell function experiments were subsequently performed. Cell proliferation was promoted by SERPINE1 overexpression while suppressed by miR‐1275 mimics (*P* < .01, Figure 5B). SERPINE1 reduced cell apoptosis, while it was remarkably enhanced by miR‐1275 mimics (*P* < .01, Figure 5C). Parallelly, cell migration (Figure 5D) and invasion (Figure 5E) were facilitated by SERPINE1 overexpression while reduced by miR‐1275 mimics (*P* < .05). In addition, co‐transfection of pcDNA3.1‐SERPINE1 and miR‐1275 mimics showed tiny changes in cell functions compared with the NC group. These results confirmed the hypothesis that miR‐1275 affected glioma cell function via regulating SERPINE1.

**Figure 5:** MiR‐1275 targeted SERPINE1 to suppress glioma cell proliferation, invasion and migration whereas enhance apoptosis. A, SERPINE1 mRNA expression was increased after pcDNA3.1‐SERPINE1 transfection while decreased after miR‐1275 mimics transfection. There was no significant difference between the expression of SERPINE1 mRNA in the NC group and miR‐1275 mimics + pcDNA3.1‐SERPINE1 group (Mix group). B, Cell proliferation of pcDNA3.1‐SERPINE1 group was highest, then the NC group and miR‐1275 mimics + pcDNA3.1‐SERPINE1 group (Mix group) followed and it was lowest in miR‐1275 mimics group. C, Cell apoptosis rate in pcDNA3.1‐SERPINE1 group was lower than those in the NC group, while that in miR‐1275 mimics group was significantly higher. Mix group showed tiny changes. D, Closed wound area in pcDNA3.1‐SERPINE1 group was larger while miR‐1275 mimics group was smaller than that in the NC group. Mix group showed tiny changes. E, Number of invasive cells in pcDNA3.1‐SERPINE1 group was the highest while it was lowest in miR‐1275 mimics group. There was no significant difference between Mix group and NC group. *P < .05, **P < .01, compared with the NC group

### 3.6 MiR‐1275 blocked p53 signalling pathway

Effect of miR‐1275 and SERPINE1 on expression of p53 pathway‐associated proteins was detected by western blot. Since U251 was p53 mutant‐type, we performed the experiment using both U251 (Figure 6A) and a p53 wild‐type expressing cell line H4 (Figure 6B). Moreover, we used a p53 signalling pathway agonist RITA (NSC 652287, MedChemExpress, Monmouth Junction, NJ, USA), which was considered to have the ability of activating wild‐type p53 to explore the effect of miR‐1275/SERPINE1 on p53 signalling pathway. The results showed that several p53 pathway‐associated proteins p21, Bax and cleaved Caspase3 were lowly expressed in both p53 wild‐type and mutant‐type expressing cells (H4/U251). After RITA (1 mmol/L) treatment, p21, Bax and cleaved Caspase3 were significantly up‐regulated in H4 cells (*P* < .05) but there was no remarkable change in U251 cells. However, SERPINE1 overexpression or miR‐1275 inhibitor significantly reduced the expressions of p21, Bax and cleaved Caspase3 in both H4 and U251 cells, while miR‐1275 mimics had inverse effects (*P* < .05). These results suggested that miR‐1275/SERPINE1 repressed p53 signalling pathway, and this effect might not be directly associated with the mutation status of TP53 gene.

**Figure 6:** MiR‐1275 promoted the expression of p53 pathway‐associated proteins. A, Western blot of U251 cells: expressions of p21, Bax and cleaved Caspase3 were not significantly changed after RITA (1 mmol/L) treatment while they were up‐regulated by miR‐1275 mimics and down‐regulated by pcDNA3.1‐SERPINE1 or miR‐1275 inhibitor. A, Western blot of H4 cells: expressions of p21, Bax and cleaved Caspase3 were up‐regulated by miR‐1275 mimics. B, RITA treatment and down‐regulated by pcDNA3.1‐SERPINE1 or miR‐1275 inhibitor. *P < .05, **P < .01, compared with the NC group

### 3.7 MiR‐1275 suppressed glioma growth in vivo

Tumour xenograft model was built to test the effect of miR‐1275 and SERPINE1 on tumour growth in vivo. Injection of agomir‐1275 and lentiviral sh‐SERPINE1 showed a parallel result that tumour volume and weight were significantly lower than the NC group (*P* < .01, Figure 7A‐C). Tumour tissues were collected and immunohistochemistry was performed to detect tumour‐related proteins. Compared with the NC group, p53 and cleaved Caspase3 positive rate was higher, whereas MDM2 and ki67 positive rate was lower in agomir‐1275 and sh‐SERPINE1 groups (Figure 7D). Based on these results, we reach the conclusion that miR‐1275 overexpression or SERPINE1 silencing would suppress glioma growth.

**Figure 7:** MiR‐1275 promoted glioma growth in vivo. A, Tumour specimens’ images. B, Tumour volumes of agomir‐1275 group and sh‐SERPINE1 group were decreased compared with the NC group. C, Tumour weights of agomir‐1275 group and sh‐SERPINE1 group were lower than those of NC group. D, Immunohistochemistry results of mice tumour tissues: expressions of p53 and cleaved Caspase3 were increased while expression of SERPINE1, MDM2 and ki67 was decreased in agomir‐1275 group and sh‐SERPINE1 group. **P < .01, compared with the NC group

## 4 DISCUSSION

In our study, it was revealed that lowly expressed miR‐1275 in glioma could repress glioma cell proliferation, migration and invasion whereas induce cell apoptosis through targeting SERPINE1, which was aberrantly overexpressed in glioma. Furthermore, we found that several key proteins related to p53 signalling pathway were activated by miR‐1275 while repressed by SERPINE1, revealing that the effect of miR‐1275/SERPINE1 might be based on regulating p53 signalling pathway.

Glioma is the most common and invasive type of major brain tumour, with a high yearly mortality rate worldwide.^19^, ^20^ It has now been clearly established that miRNAs have an important role to regulate the tumorigenesis and metastasis of glioma.^21^, ^22^ MiR‐1275 is an intergenic miRNA, which is encoded by chromosome 6 and associated with tumour progression.^23^ In many researches, miR‐1275 was found to inhibit tumour growth through attenuating relative gene expression. For instance, up‐regulation of miR‐1275 regulated IGF2BPs to hinder tumour growth in hepatocellular carcinoma.^24^ It was reported that miR‐1275 exhibited its tumour suppressive role on nasopharyngeal carcinoma cells by down‐regulating oncogenic HOXB5, whose expression was negatively related to miR‐1275.^25^ In our study, we found that miR‐1275 was lowly expressed in glioma and its up‐regulation could suppress glioma cell function including proliferation, migration and invasion, as well as induce apoptosis. Our discovery was consistent with the generally reported conclusion that miR‐1275 works as a tumour suppressor. However, it was reported that Katsushima et al^11^ found that inhibition of miR‐1275 increased the expression of CLDN11 with a specific antisense oligonucleotide (anti‐miR‐1275) in GSCs and also suppressed tumour growth. It indicated that the function of miR‐1275 varied in glioma and glioma stem cells.

As mentioned above, miRNAs usually exert their functions of controlling tumour growth through binding to their target genes. In our study, we found that miR‐1275 could bind to SERPINE1, which was highly expressed in glioma. Clinically, SERPINE1 and its family member urokinase‐type plasminogen activator (uPA) both have been considered as important prognostic markers for various cancers, including breast cancer^26^ and papillary thyroid cancer.^27^ Our study further confirmed that it worked as a tumour promotor in glioma.

We also found that p53 signalling pathway might participate in the development of glioma. As a major tumour suppressor, p53 can be activated by a number of cellular stressors, including DNA damage, hypoxia and oncogene activation to impact the progression of various cancers distinctly.^28^, ^29^ P53 mutation has been reported in about 30%‐50% of gliomas and it was strongly associated with the poor prognosis of glioma patients.^30^ On the other hand, wild‐type p53 could repair the cells even with genetic abnormalities^31^ and might cause drug resistance to temozolomide.^32^ SERPINE1 was generally considered as the downstream gene of p53 and could be induced by the activation of p53.^33^, ^34^ However, our study found that the up‐regulation of SERPINE1 repressed p53 signalling pathway, whereas miR‐1275 had an inverse effect, which has not been reported in previous studies. It revealed the possibility of SERPINE1′s feeding back to its upstream genes and negatively regulating p53 signalling pathway. However, the detailed molecular mechanism of this axis needs to be further explored.

## 5 CONCLUSION

In our study, we elucidated the function of miR‐1275 on glioma that it suppressed proliferation, migration, invasion and induced apoptosis in glioma. We further investigated that highly expressed SERPINE1 was a target gene of miR‐1275, and miR‐1275 exerted its tumour suppressing function through blocking SERPINE1. Moreover, we found that p53 signalling pathway was involved in this process and it could be repressed by SERPINE1 or activated by miR‐1275. Hence, we concluded that miR‐1275 worked as a tumour suppressor through binding to SERPINE1 and therefore activating p53 signalling pathway in glioma. This discovery provided a new biomarker and offered a novel potential strategy in the diagnosis and treatment of glioma.

## DECLARATIONS

## ETHICS APPROVAL AND CONSENT TO PARTICIPATE

N/A.

## CONSENT FOR PUBLICATION

This manuscript has been approved by all authors for publication.

## AVAILABILITY OF DATA AND MATERIAL

N/A.

## CONFLICT OF INTEREST

No conflict of interest exits in the submission of this manuscript.

## AUTHORS’ CONTRIBUTIONS

Substantial contribution to the conception and design of the work: Dong‐Mei Wu, Shan Wang, Xin Wen & Xin‐Rui Han; analysis and interpretation of the data: Yong‐Jian Wang, Shao‐Hua Fan, Zi‐Feng Zhang & Qun Shan; drafting the manuscript: Dong‐Mei Wu & Shan Wang; revising the work critically for important intellectual content: Jun Lu & Yuan‐Lin Zheng; final approval of the work: all authors.
